# An Immunohistochemical Study of the Increase in Antioxidant Capacity of Corneal Epithelial Cells by Molecular Hydrogen, Leading to the Suppression of Alkali-Induced Oxidative Stress

This article has been retracted.

**DOI:** 10.1155/2020/7435260

**Published:** 2020-06-21

**Authors:** Cestmir Cejka, Jan Kossl, Vladimir Holan, John H. Zhang, Jitka Cejkova

**Affiliations:** ^1^Institute of Experimental Medicine of the Czech Academy of Sciences, Vídenska 1083, 14220 Prague 4, Czech Republic; ^2^Faculty of Natural Science, Charles University, Vinicna 7, 12843 Prague 2, Czech Republic; ^3^Loma Linda University School of Medicine, Loma Linda, CA 92350, USA

## Abstract

Corneal alkali burns are potentially blinding injuries. Alkali induces oxidative stress in corneas followed by excessive corneal inflammation, neovascularization, and untransparent scar formation. Molecular hydrogen (H_2_), a potent reactive oxygen species (ROS) scavenger, suppresses oxidative stress and enables corneal healing when applied on the corneal surface. The purpose of this study was to examine whether the H_2_ pretreatment of healthy corneas evokes a protective effect against corneal alkali-induced oxidative stress. Rabbit eyes were pretreated with a H_2_ solution or buffer solution, by drops onto the ocular surface, and the corneas were then burned with 0.25 M NaOH. The results obtained with immunohistochemistry and pachymetry showed that in the corneas of H_2_-pretreated eyes, slight oxidative stress appeared followed by an increased expression of antioxidant enzymes. When these corneas were postburned with alkali, the alkali-induced oxidative stress was suppressed. This was in contrast to postburned buffer-pretreated corneas, where the oxidative stress was strong. These corneas healed with scar formation and neovascularization, whereas corneas of H_2_-pretreated eyes healed with restoration of transparency in the majority of cases. Corneal neovascularization was strongly suppressed. Our results suggest that the corneal alkali-induced oxidative stress was reduced via the increased antioxidant capacity of corneal cells against reactive oxygen species (ROS). It is further suggested that the ability of H_2_ to induce the increase in antioxidant cell capacity is important for eye protection against various diseases or external influences associated with ROS production.

## 1. Introduction

A corneal alkali injury often causes extensive damage to the ocular surface and the whole anterior eye segment, leading to permanent vision impairment or even complete blindness. Immediately following a severe injury, such as corneal alkali burn or the repeated ultraviolet (UVB) irradiation of corneas, oxidative stress occurs in the corneas. In corneal epithelial cells, an antioxidant/prooxidant imbalance appears [1–7]. Reactive oxygen species (ROS) which have been insufficiently cleaved greatly contribute to excessive intracorneal inflammation and corneal healing with scar formation and neovascularization [4].

Molecular hydrogen (H_2_), a cleaving reactive oxygen species (ROS), dissolved in buffer and applied onto the corneal surface after the alkali injury, suppresses corneal oxidative stress which prevents the development of excessive inflammation and corneal neovascularization [4, 6, 7]. H_2_ cleaves hydroxyl radicals and peroxynitrite, which react with nucleic acids, lipids, and proteins, resulting in deoxyribonucleic acid (DNA) fragmentation, lipid peroxidation, and protein inactivation [8, 9]. H_2_ can diminish oxidative stress and effectively reduce the active ROS that are associated with diseases. H_2_ does not affect the ROS required for physiological functions. Despite their cytotoxic effects, low concentrations of ROS, such as superoxide and hydrogen peroxide, function as signaling molecules and regulate apoptosis, cell proliferation, and differentiation. As H_2_ reduces hydroxyl radicals but does not affect superoxide and hydrogen peroxide having physiological roles, it is proposed that the adverse effects of H_2_ are very small compared to those of other antioxidants [10–12]. Murakami et al. [13] described how H_2_ can act not only as a free radical scavenger but also as a mitohormetic effector against oxidative stress in cells. The authors found that the pretreatment of cultured neuroblastoma SH-SY5Y cells with H_2_ suppressed H_2_O_2_-induced cell death. In H_2_-treated cells, the expression of antioxidant enzymes was increased, indicating that H_2_ induced mild stress and increased the resistance to exacerbated oxidative stress. According to Iketani et al. [14], the pretreatment of mice by drinking H_2_ water for three days protected them against lipopolysaccharide- (LPS-) induced sepsis and attenuated liver injury. H_2_ water was able to trigger an adaptive response against oxidative stress.

In this study, H_2_ dissolved in a buffer or buffer H_2_-free solution was dropped onto the corneal surface of healthy rabbit eyes and then, the eyes were postburned with alkali. In postburned H_2_-pretreated eyes, the alkali-induced oxidative stress was reduced. As the pretreatment of eyes with H_2_ induced slight oxidative stress in the corneal epithelium, followed by the increased expression of antioxidant enzymes, it is suggested that the alkali-induced oxidative stress was suppressed through the increased antioxidant capacity of corneal epithelial cells against ROS.

## 2. Materials and Methods

### 2.1. Preparation of H_2_ Saturated in Phosphate-Buffered Saline (PBS)

Original Dr. Hidemitsu Hayashi's HydrogenRich Water Stick and original Dr. Hayashi Glass Bottle (The HydrogenRich Water Group LLC Lawrence, KS, USA) were used as previously described [6, 7]. Briefly, the special glass bottle was filled with the PBS and the hydrogen stick was immersed into the bottle. The bottle was tightly closed without the dead volume. The bottle was shaken for 15 seconds and left to stand for 20 minutes. The stick was then removed from the bottle. The small amount of missing solution was refilled with PBS, and the bottle tightly closed.

### 2.2. Measuring H_2_ Concentration in PBS Solution

For the measurement of H_2_ concentration in PBS, the Unisense H_2_ Microsensor was used. This microsensor is the Clark-type sensor measuring hydrogen partial pressure. The resulting sensor signal is in the picoammeter (pA) current range. This signal is measured by the Unisense Microsensor Multimeter. The multimeter readings can be transferred (according to the manual of the multimeter) to the concentrations of the dissolved H_2_ in PBS in mmol/L. According to Ohta [10], H_2_ can be dissolved in water up to 1.6 ppm wt/vol (0.8 mM) under atmospheric pressure. In our study, the H_2_ concentration measured immediately after preparing the solution was 1.5 ± 0.2 pulse position modulation (ppm) weight/volume, showing that the H_2_ solution was saturated (for details, see [6, 7]).

### 2.3. Experimental Animals

Adult female New Zealand white rabbits (2.5-3.0 kg) were used in our experiments. The investigation was conducted according to the ARVO Statement on the Use of Animals in Ophthalmic and Vision Research. The experiments were approved by the local ethics committee of the Institute of Experimental Medicine under the No. 123/2016.

### 2.4. The Pretreatment of Eyes with H_2_ (H_2_ Dissolved in PBS) or Buffer (PBS-H_2_-Free Solution)

The right eyes of fifteen rabbits were pretreated with a H_2_ solution in one group of animals and with a buffer solution in the other group of animals (fifteen rabbits), before the corneal alkali burns. The pretreatment took place by applying five drops of H_2_ solution or buffer solution four times daily, onto the ocular surface, for three days. Five rabbits from each group were sacrificed, and the corneas were investigated for ROS and antioxidant enzymes. The other pretreated animals were used for corneal alkali burn.

### 2.5. The Alkali Injury of Corneas in Experimental Animals

The rabbits (ten animals from each group of pretreated eyes) were anesthetized by an intramuscular injection of Rometar (xylazinum hydrochloricum, Spofa, Prague, CR, 2%, 0.2 mL/kg body weight) and Narkamon (ketaminum hydrochloricum, Spofa, 5%, 1 mL/kg body weight). Sodium hydroxide (0.25 M NaOH) was applied by means of dropping on the corneal surface (10 drops during 1 minute) of H_2_-pretreated eyes or buffer-pretreated eyes. The eyes were then irrigated with tap water. Five rabbits from each group were sacrificed, and the eyes examined for ROS by dihydroethidium (DHE) assay and for the immunohistochemical examination of antioxidant enzymes. The other rabbits (the remaining five animals from each group) were left without any treatment until the end of the experiment (day 23).

After the alkali injury and awakening from anesthesia, the rabbits were treated with analgesia (ketoprofen, 1.0 mg/kg i.m.) twice daily for five days. The animals were sacrificed following an i.v. injection of thiopental anesthesia (thiopental, Spofa, 30 mg/kg), after premedication with an intramuscular injection of Rometar/Narkamon. In all of the experiments with an alkali injury, the corneas of healthy rabbit eyes served as the controls. Photographs of the corneas were taken throughout the whole experiment.

### 2.6. Dihydroethidium (DHE) Assay

The eyes were enucleated and immediately quenched in light petroleum chilled with an acetone-dry ice mixture. Sections were cut on a cryostat and transferred to glass slides. Unfixed cryosections (10 *μ*m) were incubated with 5 *μ*M DHE (Sigma-Aldrich, St. Louis, MO, USA) for 15 minutes at 37°C. A negative control was created by incubating sections with PBS instead of DHE. Sections were examined using a microscope equipped with a digital camera (Leica, Germany), and the intensity of the staining was measured using the Fiji ImageJ Program [15].

### 2.7. Immunofluorescence Staining

After sacrificing the animals, the eyes were enucleated, and the anterior eye segments dissected and quenched in light petroleum chilled with an acetone-dry ice mixture. Sections were cut on a cryostat and transferred to glass slides. Subsequently, the cryostat sections were fixed in acetone at 4°C for 5 minutes. For the detection of MDA, NT, and iNOS, the postfixed cryostat sections (in acetone at 4°C for 5 minutes) were incubated (60 minutes) with monoclonal mouse anti-iNOS (Biosciences, San Jose, CA, USA) or monoclonal mouse anti-NT (Abcam, Cambridge, UK) or polyclonal goat anti-MDA (US Biological, Swampscott, MA, USA), followed by 45 min incubation by Alexa Fluor 488 Goat Anti-Mouse IgG or Alexa Fluor 488 Donkey Anti-Goat IgG (Thermo Fisher Scientific, Waltham, MA, USA). Following the procedure, the samples were immediately examined using the microscope Leitz (Orthoplan Leitz light microscope equipped with a Leica DC 500 digital camera).

### 2.8. Immunohistochemical Staining

Postfixed cryostat sections in acetone (at 4°C for 5 minutes) were used. For vascular endothelial growth factor (VEGF) and matrix MMP 9, CAT, and SOD, the following primary antibodies were used: rabbit polyclonal anti-SOD-1 (Abcam), rabbit polyclonal anti-CAT (Abcam), mouse monoclonal anti-VEGF (Abcam), and goat polyclonal anti-MMP 9 (Santa Cruz Biotechnology, Santa Cruz, California, USA). The binding of the primary antibodies was demonstrated using the HRP/DAB UltraVision Detection System, as described previously (6,7). For secondary antibodies, biotinylated goat anti-rabbit IgG, biotinylated goat anti-mouse IgG, or donkey anti-goat IgG (Thermo Fisher Scientific) (10 minutes) were employed. Cryostat sections in which the primary antibodies were omitted from the incubation media, served as negative controls. The sections for VEGF and MMP9 were counterstained with Mayer's hematoxylin. After the staining procedure, the samples were immediately examined using an Orthoplan Leitz light microscope, equipped with a Leica DC 500 digital camera.

### 2.9. Determination of Corneal Thickness

Changes in the levels of corneal thickness after the injury and during healing were evaluated by measuring the central corneal thickness (taken as an index of corneal hydration) (see Cejka et al. [16] in detail). Briefly, the central corneal thickness was measured in anesthetized animals using an ultrasonic pachymeter SP-100 (Tomey Corporation, Nagoya, Japan) in the corneal center. The corneal thickness was measured in the same corneas before H_2_ or buffer pretreatment and alkali injury (corneas of healthy eyes), and then, two, ten, and twenty days after the injury (all experimental groups). Each cornea was measured four times, and the mean and standard deviation of the thickness (in *μ*m) were computed.

### 2.10. The Evaluation of Corneal Neovascularization

For the evaluation of corneal neovascularization, the number of vessels was counted in each 60° sector of the corneal surface (see Cejkova et al. [17] in detail). The mean value and standard deviation were counted from five measurements.

### 2.11. Statistical Analysis

The analysis of the data showed normal distribution, and the results are expressed as mean ± SD. Comparisons between two groups were made by the Student *t*-test, and multiple comparisons were analyzed by ANOVA. A value of *p* < 0.05 was considered statistically significant. For corneal thickness, paired *t*-test was employed.

## 3. Results

### 3.1. Graphical Schemes of the Course of Experiment with H_2_ (Dissolved in Buffer, PBS) or with Buffer (PBS-H_2_-Free Solution) Are Shown in Figure 1

#### 3.1.1. Groups of Experimental Animals

In our study, there were three groups of rabbits: the group with alkali-injured corneas pretreated with H_2_, the group with alkali-injured corneas pretreated with buffer, and the group of animals with alkali-injured corneas of unpretreated eyes. The results of the injured corneas of unpretreated eyes did not differ from the results obtained from the injured corneas of eyes pretreated with buffer (H_2_-free). For this reason, the results of the alkali-injured unpretreated group are not shown.

### 3.2. The ROS Production and Antioxidant Enzyme Expression in Corneas of H_2_- or Buffer-Pretreated Eyes

The application of H_2_ dissolved in buffer (0.8 ppm) on the corneal surface of healthy eyes four times daily for three days induced the increase in ROS expression in the corneal epithelium (mild oxidative stress shown using DHE assay). The mild oxidative stress was accompanied with the increased expression of antioxidant enzymes in the corneal epithelium, shown with superoxide dismutase (SOD) and catalase (CAT) expressions. Macroscopically, no changes are seen on the buffer-pretreated eyes, as well as the H2-pretreated eyes, compared to the controls (Figure 2). The rabbits were sacrificed after the three-day pretreatment of eyes with H_2_ or buffer, and the corneas examined.

### 3.3. The Corneal Alkali-Induced Oxidative Stress in the Corneas of Eyes Pretreated with H_2_ or Buffer

In the control corneal epithelium, ROS production is low and SOD and CAT expressions of significant levels are present. Compared to the controls, the increased ROS production is seen in the alkali-injured corneal epithelium of eyes pretreated with buffer, whereas the expressions of SOD and CAT are strongly decreased. In contrast to these eyes, the ROS production in the corneal epithelium of eyes pretreated with H_2_ and alkali injured is low and the expressions of SOD and CAT are less decreased, compared to the alkali-injured buffer-pretreated eyes (Figure 3). This corresponds with the macroscopical picture of corneas. The alkali-injured corneas of buffer-pretreated eyes are swollen and untransparent (Figure 3).

### 3.4. The Expression of Malondialdehyde (MDA), Nitrotyrosine (NT), Inducible Nitric Oxide Synthase (iNOS), Vascular Endothelial Growth Factor (VEGF), and Matrix Metalloproteinase 9 (MMP 9) in Alkali-Injured Corneas of Eyes Pretreated with H_2_ or Buffer

The expression of MDA (a marker of oxidative stress), peroxynitrite (a marker of lipid peroxidation, detected by NT residues), iNOS, MMP 9, and VEGF was increased in the alkali-injured corneas of buffer-pretreated eyes, whereas in the alkali-injured corneas of H_2_-pretreated eyes, the expressions were low or almost absent (Figure 4). In order to reveal the structure of the cornea, VEGF and MMP 9 expressions were shown with immunohistochemical staining (HRP/DAB), and sections were counterstained with hematoxylin. It can be shown that in alkali-injured corneas of buffer-pretreated eyes, the epithelium is absent or the corneas are covered with a thin and irregular epithelium. The corneas are then vascularized. The animals were sacrificed at the end of the experiment.

### 3.5. The Macroscopical Picture of Corneas and the Central Thickness of Corneas (Taken as an Index of Corneal Hydration) of Eyes Pretreated with H_2_ or Buffer

The macroscopical picture shows that the alkali-injured corneas of H_2_-pretreated eyes heal with the restoration of transparency, whereas the corneas of buffer-pretreated eyes heal with neovascularization and scar formation (Figure 5(a)). Four hours after the alkali injury of the eyes pretreated with buffer, the levels of corneal hydration are more elevated than the levels of corneal hydration of the eyes pretreated with H_2_ (Figure 5(b)). Subsequent levels of corneal hydration of the buffer-pretreated eyes were highly elevated during the experiment, and they did not reach the levels prior to injury until the end of the experiment. In contrast, in the H_2_-pretreated eyes, the corneal hydration was less increased during the experiment and it finally reached the levels before injury (Figure 5(c)).

### 3.6. Corneal Neovascularization in the Alkali-Injured Corneas of H_2_- or Buffer-Pretreated Eyes

The corneal neovascularization was significantly suppressed in the alkali-injured corneas of H_2_-pretreated eyes, compared with the alkali-injured corneas of buffer-pretreated eyes, where the corneal neovascularization was apparent (Figure 5(d)).

## 4. Discussion

H_2_ has displayed multiple functions, including antioxidant, anti-inflammatory, antiapoptotic, and antiallergic activities [18–20]. H_2_ regulates various signal transduction pathways and the expression of various genes [11]. For these important activities, particularly antioxidant, H_2_ has proved to be effective in the treatment of diseases of various organs and tissues, such as the eye, brain, spinal cord, ear, lung, heart, liver, kidney, pancreas, intestine, muscle, and cartilage [12, 18, 21–24], in which oxidative stress was involved. For ocular diseases, associated with excessive ROS production and H_2_ treatment, particular attention has been devoted to retinal diseases. H_2_ showed neuroprotective effects in retinal ischemia-reperfusion injury [25] and a protective effect against blue light-induced retinal damage [26]; a H_2_-rich saline protected the retina against glutamate excitotoxic injury [27], H_2_ therapeutically influenced the retinopathy induced by hypoxia [28], and ameliorated the retina against light-induced damage [29]. Tao et al. [30] described H_2_ treatment as a novel strategy against photoreceptor degeneration in retinitis pigmentosa patients.

In the anterior eye segment, chemical injury or the irradiation of corneas with UVB rays induces severe corneal injury, which was favorably influenced by H_2_ treatment [4, 6, 7]. A chemical injury of the cornea in humans caused by various toxic chemicals, particularly alkalis, often occurs in industry and in the household. The alkali quickly penetrates through the cornea into the deeper parts of the eye. Irradiation of the cornea with UVB rays causes photodamage. Both injuries are very dangerous to the eye. The oxidative stress appears in the corneas immediately after the alkali or UVB irradiation injury [4, 6, 7]. In the corneal epithelium, an antioxidant/prooxidant imbalance appears [1, 3], followed by a protease/antiprotease imbalance [31, 32] and proinflammatory cytokine induction [3, 33]. This leads to excessive inflammation, corneal ulceration, or healing with scar formation and neovascularization [3, 4]. The vision is partially or totally lost. H_2_ dissolved in buffer, applied immediately or very early after the injury on the corneal surface, suppresses oxidative stress and protects corneas against a strong inflammatory response [4, 6, 7]. This is very important for the reason that corneal inflammation is the trigger of angiogenesis after injury [4].

When comparing the previous healing results of alkali-burned corneas directly treated with H_2_ [4, 6] with the healing results in this study of H_2_-pretreated corneas postburned with alkali (Figure 1), we can summarize that in both cases, the alkali-induced oxidative stress was suppressed, which enabled corneal healing. To show these effects, similar markers of oxidative stress and lipid peroxidation, as well as corneal ultrasonic pachymetry for the measurement of the central corneal thickness taken as an index of corneal hydration [16], were employed in both cases. However, in the abovementioned studies, the mechanism of oxidative stress reduction was different. In the treatment of alkali-burned cornea with H_2_ solution dropped on the corneal surface, the direct antioxidant effect of H_2_ was observed. In the second case, in experiments with H_2_ pretreatment, the alkali-induced corneal oxidative stress was reduced through the increased antioxidant capacity of corneal cells against ROS. We believe that this paper is the first to study the preventive effect of H_2_ on the healing of ocular injuries and diseases, although Japanese authors have described this effect in nonophthalmological experimental models [13, 14].

Murakami et al. [13] investigated the effect of H_2_ on mitochondria in cultured SH-SY5Y neuroblastoma cells. The pretreatment of cells with H_2_ increased the mitochondrial membrane potential and the cellular ATP level, which were accompanied by a decrease in the reduced glutathione level and an increase in the superoxide level. The H_2_ pretreatment of cells prevented H_2_O_2_-induced cell death and enhanced mitochondrial activities; this was accompanied by an increased level of oxidative stress, and it then induced the increased expression of antioxidant enzymes. According to these authors, H_2_ can protect cells against oxidative stress, not only as an ROS scavenger but also as a mitohormetic effector.

Iketani et al. [14] in a mouse model of sepsis pretreated animals with H_2_ by administering H_2_ water for three days before LPS injection. The H_2_ pretreatment reduced both the apoptosis of liver cells and oxidative stress. Moreover, the pretreatment enhanced the LPS-induced expression of heme oxygenase-1 and reduced endothelin-1 expression. The authors concluded that this indicated the therapeutic potential of H_2_ water in preventing acute injury of the liver, with attenuation of an increased oxidative stress. H_2_ water was likely to trigger adaptive responses against oxidative stress.

In our study, the H_2_ pretreatment of corneas induced mild oxidative stress in the corneal epithelium, accompanied by an increased expression of antioxidant enzymes, reducing oxidative corneal damage in postburned eyes (Figures 2–4). Our present results, along with those obtained previously [6, 7], show that H_2_ has a direct antioxidant effect by reducing ROS and also inducing the adaptive protective response against ROS.

## 5. Conclusion

Both H_2_ activities (H_2_ as the ROS scavenger and H_2_ as the adaptive response inducer against ROS, Figure 6) are very important for the healing of ocular diseases with excessive ROS production. H_2_ is able to improve diseases by ROS reduction and slowing the progression of diseases by the induction of the increased antioxidant cell resistance to ROS. H_2_ in eye drops may be very helpful in the treatment of ocular diseases, such as dry eye disease or conjunctival inflammatory disorders, both influenced by various internal and external influences, associated with ROS production.

## Figures and Tables

**Figure 1:** Graphical schemes of the course of experiment with H_2_ (H_2_ dissolved in buffer, PBS) or buffer (PBS-H_2_-free solution).

**Figure 2:** Macroscopical images of eyes and increased ROS production and antioxidant enzyme expression after H_2_ pretreatment. The animals were sacrificed after three-day pretreatment of eyes with H_2_ or buffer and the corneas examined. The production of ROS, SOD, and CAT expressions in the corneal epithelium of eyes pretreated with H_2_, is higher compared to that in the control corneal epithelium or corneal epithelium pretreated with buffer. The intensities of DHE, SOD, and CAT expressions are quantified. The values with asterisks are significantly different (^∗∗^*p* < 0.01, ^∗∗∗^*p* < 0.001) from buffer-pretreated corneas. Buffer-pretreated DHE 1.013 ± 0.115; H_2_-pretreated DHE 1.825 ± 0.023; control DHE 0.999 ± 0.091; buffer-pretreated SOD 1.006 ± 0.078; H_2_-pretreated SOD 1.652 ± 0.059; control SOD 1.003 ± 0.039; buffer-pretreated CAT 0.972 ± 0.081; H_2_-pretreated CAT 1.375 ± 0.117; control CAT 0.993 ± 0.054; *n* = 5/group. Scale bars: 50 *μ*m.

**Figure 3:** In alkali-injured corneal epithelium of H_2_-pretreated eyes, the alkali-induced oxidative stress is suppressed. The animals were euthanized immediately after corneal alkali injury, followed after three-day pretreatment of healthy eyes with H_2_ or buffer and the corneas examined. Compared to the alkali-injured corneas of buffer-pretreated eyes, where oxidative stress is strong in the corneal epithelium and expressions of antioxidant enzymes (SOD, CAT) decreased, in the alkali-injured corneal epithelium of H_2_-pretreated eyes, the oxidative stress is reduced and the expression of antioxidant enzymes is nearly at physiological levels (compared to controls). DHE, SOD, and CAT expression intensities are quantified. The values with asterisks are significantly different (^∗^*p* < 0.1, ^∗∗^*p* < 0.01, ^∗∗∗^*p* < 0.001) from the buffer-pretreated corneas. Buffer-pretreated DHE 2.397 ± 0.066; H_2_-pretreated DHE 1.491 ± 0.352; control DHE 1.000 ± 0.231; buffer-pretreated SOD 0.540 ± 0.024; H_2_-pretreated SOD 0.867 ± 0.021; control SOD 0.998 ± 0.02; buffer-pretreated CAT 0.589 ± 0.035; H_2_-pretreated CAT 0.937 ± 0.018; control CAT 0.997 ± 0.026; *n* = 5/group. Scale bars: 50 *μ*m.

**Figure 4:** The expression of malonaldehyde (MDA), nitrotyrosine (NT), inducible nitric oxide synthase (iNOS), vascular endothelial growth factor (VEGF), and matrix metalloproteinase 9 (MMP9) is high in alkali-injured corneas of buffer-pretreated eyes. The animals were euthanized at the end of experiments, and the corneas examined. MDA, NT, iNOS, VEGF, and MMP9 are expressed in cells of the corneal epithelium and corneal stroma and in cells that invaded the corneal stroma (white arrows) of alkali-injured buffer-pretreated eyes (b, e, h, k, n), whereas in the alkali-injured corneas of H_2_-pretreated eyes (c, f, i, l, o), the expressions of individual markers are almost absent. The alkali-injured corneas of buffer-pretreated eyes are vascularized (black arrows, N). Scale bars: 50 *μ*m.

**Figure 5:** A macroscopical picture of alkali-injured corneas of eyes pretreated with H_2_ or buffer on days 10 and 20 after alkali injury, the central corneal thickness, and corneal neovascularization (a). Alkali-injured corneas of eyes pretreated with H_2_ heal with the restoration of transparency. In contrast, the alkali-injured corneas of eyes pretreated with buffer heal with scar formation (b). The central corneal thickness (corneal hydration) is highly increased in the corneas of buffer-pretreated eyes, after only four hours following corneal alkali burn. This then decreases but did not reach the levels before injury until the end of the experiment (c). The corneal neovascularization was suppressed in the alkali-injured corneas of H_2_-pretreated eyes (d). Each bar represents the mean ± SD from 5 corneas. The values with asterisks are significantly different (^∗∗∗^*p* < 0.001) from the buffer-pretreated alkali-injured corneas. The values with asterisks are significantly different (^∗∗∗^*p* < 0.001) from the buffer-pretreated alkali-injured corneas.

**Figure 6:** The effect of H_2_ pretreatment of healthy corneas on alkali-induced oxidative stress in postburned eyes is shown.

## Data Availability

The data used to support the findings of this study are available from the corresponding author upon request.

## Abbreviations

H_2_: Molecular hydrogen
MMP 9: Matrix metalloproteinase 9
MDA: Malondialdehyde
NT: Nitrotyrosine
ROS: Reactive oxygen species
SOD: Superoxide dismutase
CAT: Catalase
VEGF: Vascular endothelial growth factor
DHE: Dihydroethidium
iNOS: Inducible nitric oxide synthase
LPS: Lipopolysaccharide.
